The article "Gene Position Index Mutation Detection Algorithm Based on Feedback Fast Learning Neural Network" was retracted in 2023. Reasons: signs of a paper mill; compromised peer review; unreliable results or conclusions.

# Gene Position Index Mutation Detection Algorithm Based on Feedback Fast Learning Neural Network

**DOI:** 10.1155/2021/1716182

**Published:** 2021-07-06

**Authors:** Zhike Zuo, Chao Tang, Yu Xu, Ying Wang, Yongzhong Wu, Jun Qi, Xiaolong Shi

**Affiliations:** ^1^Chongqing Key Laboratory of Spatial Data Mining and Big Data Integration for Ecology and Environment, Chongqing Finance and Economics College, Chongqing 401320, China; ^2^Radiation & Cancer Biology Laboratory, Radiation Oncology Center, Chongqing Key Laboratory of Translational Research for Cancer Metastasis and Individualized Treatment, Chongqing University Cancer Hospital & Chongqing Cancer Institute & Chongqing Cancer Hospital, Chongqing 400030, China; ^3^College of Bioengineering, Chongqing University, Chongqing, China

## Abstract

In the detection of genome variation, the research on the internal correlation of reference genome is deepening; the detection of variation in genome sequence has become the focus of research, and it has also become an effective path to find new genes and new functional proteins. The targeted sequencing sequence is used to sequence the exon region of a specific gene in cancer gene detection, and the sequencing depth is relatively large. Traditional alignment algorithms will lose some sequences, which will lead to inaccurate mutation detection. This paper proposes a mutation detection algorithm based on feedback fast learning neural network position index. By establishing a position index relationship for ACGT in the DNA sequence, the subsequence is decomposed into the position relationship of different subsequences corresponding to the main sequence. The positional relationship of the subsequence in the main sequence is determined by the positional relationship. Analyzing SNP and InDel mutations, even structural mutations, through the position correlation of sequences has the advantages of high precision and easy implementation by personal computers. The feedback fast learning neural network is used to verify whether there is a linear relationship between two or more positions. Experimental results show that the mutation points detected by position index are more than those detected by Bcftools, Freebye, Vanscan2, and Gatk.

## 1. Introduction

In recent years, the research scope of chemical genomics has gradually expanded, combining combinatorial chemistry, cell molecular biology, and genetics to form a fusion technology model, and using high-throughput screening technology to conduct data analysis from a more comprehensive perspective. It is precise because the chemical genome analyzes life sciences from a new perspective; it has a certain promotion value. During the operation of chemical genomics technology, the specificity between the small molecule compound probe and the target protein can be used as an entry point to complete gene transcription operations, gene processing operations, and translation procedures, thereby enabling in-depth regulation of specific life processes.

Currently, an index is established for DNA sequences to improve the speed of searching and matching DNA sequences. DNA target regions can generally be divided into repetitive fragments and specific fragments from the composition of the sequence. Repetitive fragments refer to the sequence in the target area where there are more repeated sequences. Literature [1] proposes Hamming distance or PFD filter to find the repetitive area, but the algorithm efficiency is low, the memory is large, and the running time is long. Literature [2] proposes to search for repetitive sequences by indexing subsequent arrays, but the efficiency is still relatively low. In the method of searching for specific fragments, the specific region segment proposed in literature [3] is composed of four bases A, G, T, and C to form an irregular sequence combination. Literature [4] studies the hash index structure of the one-way hash function and the index retrieval method to search for specific fragments and similar sequences. Literature [5] also proposed a novel solution for searching for specific DNA sequences. For the construction of the hash index structure, in DNA sequence matching [6], the commonly used fixed sequences are stored in the DNA database, and the similarity is used to evaluate whether the sequences are matched successfully. Literature [7] is applied to the index values of pattern characters and subsequence characters and matches from left to right. It stores all the index values of all characters and checks the first character of the pattern, which character appears first in the pattern as the starting matching position. Literature [8] proposes to establish index structure in DNA and protein sequences, design a multithread matching model based on DNA sequence index, match sequences of multiple tasks simultaneously and has high efficiency in DNA matching accuracy. Literature [9] proposes a hash function based on Hash-q to eliminate conflicts, providing a perfect and efficient hash value generation method. Under the condition that *q* characters of pattern and text need not be compared, Hash-q has better performance in accuracy and time compared with *Escherichia coli* and human chromosome data sets. Literature [10] applies to multiple patterns matching of DNA sequences, uses index tables for strings and patterns, and uses the count variable to count the number of occurrences of each character. The character displayed with the smallest number in the pattern is considered the first choice for comparison, and the character with the largest number in the given string is matched first. In the second part of the article, the implementation method and comparison algorithm of feedback fast learning neural network are explained. The third part describes the realization process of DNA sequence positional relationship. In the fourth part, the advantages of the proposed method are verified by experiments.

## 2. Feedback Fast Learning Neural Network and DNA Comparison Algorithm

### 2.1. Fast Learning Network (FLN)

FLN [11, 12], as a new type of double parallel and feed-forward multilayer artificial neural network, has the advantages of compact network scale, short learning and training time, strong fitting ability, and so forth. FLN consists of three layers of neurons, including input layer, hidden layer, and output layer neurons; see Figure 1.

The weight matrix from the input layer to the hidden layer is **W**_*m*×*n*_, the weight matrix from the hidden layer to the output layer is **V**_*p*×*m*_, and the weight matrix from the input layer to the output layer directly without passing through the hidden layer is **U**_*p*×*n*_. FLN network can be described by

(1) $$\begin{array}{c} \left\{\begin{array}{c} L_{m\times 1}=f\left(\theta_{m\times 1}+W_{m\times n}X_{n\times 1}\right),\\ Y_{p\times 1}=g\left(\delta_{p\times 1}+V_{p\times m}L_{m\times 1}+U_{p\times n}X_{n\times 1}\right), \end{array}\right) \end{array}$$

where *n*, *m*, and *p* are the number of neurons in the input layer, hidden layer, and output layer, respectively; **X**_*n*×1_, **L**_*m*×1_, and **Y**_*p*×1_ are the input vector, hidden layer output vector, and output layer output vector of the network, respectively; *θ*_*m*×1_ and *δ*_*p*×1_are the hidden layer threshold vector and the output layer threshold vector, respectively; and *f* and *g* are the kernel functions of the hidden layer and the output layer, respectively.

### 2.2. Feedback Fast Learning Network

FLN is a feed-forward neural network, and its output is only related to the input of the network at the current moment [13, 14] but has nothing to do with the input and output of the network at the previous moment, that is, FLN ignores the connection between the output of the system at this moment and the previous output of the system. However, for systems with large inertia or delay, the output of the model is not only related to the input at the current moment but also related to the input at the previous moments, and the input at the current moment affects the output at the following moments of the model [13, 15, 16]. Based on this, a feedback fast learning network (B-FLN) is proposed to improve the performance of FLN by adding a delayed feedback channel from output to input on the basis of FLN [17, 18]. The structure diagram of B-FLN is shown in Figure 2.

In the figure, Z^−1^ is a delayed feedback link and **B**_*m*×*p*_ is the weight of the network output **Y**(*t* − 1)to the hidden layer neurons at the previous moment. The B-FLN mathematical model is described as follows, where *T* is the current time:

(2) $$\begin{array}{c} \left\{\begin{array}{c} L_{m\times 1}\left(t\right)=f\left(\theta_{m\times 1}+W_{m\times n}X_{n\times 1}\left(t\right)+B_{m\times p}Y_{p\times 1}\left(t-1\right)\right),\\ Y_{p\times 1}\left(t\right)=g\left(\delta_{p\times 1}+V_{p\times m}L_{m\times 1}\left(t\right)+U_{p\times n}X_{n\times 1}\left(t\right)\right). \end{array}\right) \end{array}$$

For B-FLN, if the weights **W**, **B**, **V,** and **U** of the network are determined, thresholds*θ*, *δ*and *f*, *g* of any input sample **X**_*n*×1_ correspond to an output vector **Y**_*p*×1_. Generally speaking, the output layer of the three-layer network takes the linear output function, while the kernel function of the hidden layer takes the “Sigmoid” function. The weights from the input layer to the hidden layer of the B-FLN and any element of the threshold value **W**, **B**, and *θ* are initialized to random values within [0, 1].

The weights **V** and **U** and thresholds *δ* from hidden layer to output layer of B-FLN are solved by Moore–Penrose generalized inverse theory. Assuming **X**(*t* − *i*) and $\hat{Y}\left(t-i\right)\left(i=0,\ldots ,N-1\right)$ that the input and output sample sequence collected sequentially from a certain system and N is the length of the sample sequence, the predicted output **Y**_*t*_of the B-FLN model is

(3) $$\begin{array}{c} \left\{\begin{array}{c} L_{t}=f\left(\mathrm{\theta I}+WX_{t}+B{\hat{Y}}_{t-1}\right),\\ Y_{t}=g\left(\mathrm{\delta I}+VL_{t}+UX_{t}\right), \end{array}\right) \end{array}$$

where **I**=[1,1,…,1]_1×*N*_.

Minimize predicted **Y**_*t*_and true values${\hat{Y}}_{t}$:

(4) $$\begin{array}{c} \left\|g\left(\left[\hat{U},\hat{V},\delta \right]\left[\begin{array}{c} X_{t}\\ Y_{t}\\ I \end{array}\right]\right)-{\hat{Y}}_{t}\right\|=\underset{U,V,\delta }{\min}\left\|Y_{t}-{\hat{Y}}_{t}\right\|. \end{array}$$

B-FLN weight and threshold determined by Moore–Penrose generalize inverse:

(5) $$\begin{array}{c} \left[\hat{U},\hat{V},\delta \right]=g^{-1}\left({\hat{Y}}_{t}\right){\left[\begin{array}{c} X_{t}\\ Y_{t}\\ I \end{array}\right]}^{†}, \end{array}$$

where the superscript symbol “†” represents the M-P generalized inverse of the matrix.

The predicted output **Y**_*t*_ of the B-FLN network can be described as a function of **X**_*t*_ and **Y**_*t*−1_, and **Y**_*t*−1_ can be described as a function of **X** _*t*−1_ and **Y** _*t*−2_. Therefore, B-FLN actually establishes the mapping relationship from sequence **X**_*t*_, **X**_*t*−1_ to **Y**_*t*_. The learning training of the B-FLN network is carried out by using the collected data samples, and the weights and thresholds of the network are determined. The steps are as follows:

1. Randomly initialize the weights **W** and **B** and threshold vector *θ*
2. The predicted value **Y**_*t*_ is calculated by using equation (3)
3. The weights **V** and **U** and the threshold vector *δ* are calculated using equation (4)

### 2.3. DNA Comparison Algorithm

The dynamic programming algorithm was also used in the DNA sequence alignment algorithm in the early days, which is a global alignment algorithm. The Needleman–Wunsch algorithm proposed by Satra et al. [19] was first used in biological sequence alignment algorithms. It has been widely used in many fields [20–22]. The basic idea of the dynamic programming algorithm is to score a given sequence, taking the sequence *S* = “ACGTACAAAT,” *T* = “ACGGTAG” as an example, as shown in the following formula:

(6) $$\begin{array}{c} \phi \left(S^{\prime }\left[i\right],T^{\prime }\left[j\right]\right)=\left\{\begin{array}{cc} +1, & S^{\prime }\left[i\right]=T^{\prime }\left[j\right],\\ 0, & S^{\prime }\left[i\right]\neq T^{\prime }\left[j\right],\\ -1, & S^{\prime }\left[i\right]=-\text{ or }T^{\prime }\left[j\right]=-. \end{array}\right) \end{array}$$

**Step 1 .**

Initialize the sequence alignment matrix.

Construct (|*S*|+1) × (|*T*|+1) initialization matrix *V*, as shown in the following formula:

(7) $$\begin{array}{c} \left\{\begin{array}{c} V\left(0,0\right)=0,\\ V\left(i,0\right)=V\left(i-1,0\right)+\phi \left(S^{\prime }\left[i\right],-\right),\;1\leq i\leq \left|S\right|,\\ V\left(0,j\right)=V\left(0,j-1\right)+\phi \left(-,T^{\prime }\left[j\right]\right),\;1\leq i\leq \left|T\right|. \end{array}\right) \end{array}$$

To initialize the matrix *V*, the effect is shown in Figure 3.

**Step 2 .**

Fill the matrix.

The current matrix value is equal to the maximum value among diagonal, horizontal, and vertical positions, and the matrix is filled numerically by the following formula:

(8) $$\begin{array}{c} V\left(i,j\right)=\max\left\{\begin{array}{c} V\left(i-1,j-1\right)+\phi \left(S^{\prime }\left[i\right],T^{\prime }\left[j\right]\right),\\ \begin{array}{c} V\left(i-1,j\right)+\phi \left(S^{\prime }\left[i\right],-\right),\\ V\left(i-1,j\right)+\phi \left(-,T^{\prime }\left[j\right]\right). \end{array} \end{array}\right) \end{array}$$

After formula (8) to fill the matrix Figure 1, the effect is shown in Figure 4.

**Step 3 .**

Backtracking on the matrix

The optimal backtracking position for the global sequence alignment is the maximum value of *V* (|*S*|, |*T*|) in the lower right corner of the matrix; from the diagonal, vertical, and horizontal directions of *V* (|*S*|, |*T*|) to *V* (0, 0), mark the optimal global path with the identifier “⟶,” and finally form the optimal global path. The effect is shown in Figure 5.

After optimization according to the path, the global optimal alignment sequence is obtained and the effect is shown in Figure 6.

## 3. Construction Method Based on the Location Index Topology Map Path

### 3.1. DNA Sequence Position Index

For a given target DNA sequence *S* and subsequence *T*, use |*S*| to denote the length of *S* and |*T*| to denote the length of *T*.

In the DNA sequence *S*, which is all composed of A, C, G, and T, the positions of the four bases are solved, {“AAAA,” “AAAC,” “AAAG,”...,“TTTT”} for a total of 256 kinds of combination. Find all the positions of each combination in DNA, similar to the index in BWT [23, 24], and its structure is shown in Figure 7.

In Figure 7, *P*_1_^1^ represents the first position of the sequence “AAAA” in the DNA, and *P*_*n*_1__^1^represents the *n*_1_ position of the sequence “AAAA” in the DNA. *n*_1_, *n*_2_, ..., *n*_256_ are not equal, and the number of positions of each sequence in DNA is not the same. *P*_1_^1^ points to *P*_1_^2^, which means that, in the DNA position structure relationship, *P*_1_^1^ is in front of *P*_1_^2^ and the position relationship is close together.

**Theorem 1 .**

Each subsequence in the DNA sequence *S* can be described by each position relationship, and the number of all positions is equal to |*S*|:

(9) $$\begin{array}{c} S=P_{1}^{1}⟶P_{2}^{2}⟶P_{3}^{255}⟶P_{ni}^{j}\cdots ⟶P_{nk}^{l},\;i,k,l=1,2,3,\ldots ,256,\\ n_{1}+n_{2}+n_{3}+\cdots +n_{256}=|S|-3. \end{array}$$

**Proof**

Suppose *S* = “*a*_1_*a*_2_*a*_3_*a*_4_…*a*_*n*_,” |*S*| = *n*, *a*_*i*_ ∈ {*A*, *C*, *G*, *T*}. Divide *S* into a sequence of four characters, namely, “*a*_1_*a*_2_*a*_3_*a*_4_,” “*a*_2_*a*_3_*a*_4_*a*_5_,” “*a*_3_*a*_4_*a*_5_*a*_6_,”…,“*a*_*n* − 3_*a*_*n* − 2_*a*_*n* − 1_*a*_*n*_” form. The possible positional relationship of *P* (“*a*_1_*a*_2_*a*_3_*a*_4_”) is described as {1, 8, 51,…, *n*_1_}, the position of *P* (“*a*_2_*a*_3_*a*_4_*a*_5_”) is {3, 9, 10,…, *n*_2_}, and the positional relationship of *P* (“*a*_3_*a*_4_*a*_5_*a*_6_”) is described as {4, 12, 98,…, *n*_3_}; then, *P* (“*a*_*n* − 3_*a*_*n* − 2_*a*_*n* − 1_*a*_*n*_”) represents the position {43, 98,…, *n*_*n* − 3_}. Let *P*_1_^1^ = {1, 8, 51,…, *n*_1_}, *P*_2_^2^ = {2, 9, 10,…, *n*_2_}, and *P*_*nk*_^*l*^ = {43, 98,…, *n*_*n* − 3_}.

If *P* (“*a*_1_*a*_2_*a*_3_*a*_4_”) ∩ {*P* (“*a*_2_*a*_3_*a*_4_*a*_5_”) − 1} = {1, 8, 51,…, *n*_1_} ∩ {{2, 9, 10,…, *n*_2_} − 1} ≠ Φ, then *P*_1_^1^ ⟶ *P*_2_^2^.

If *P* (“*a*_2_*a*_3_*a*_4_*a*_5_”) ∩ {*P* (“*a*_3_*a*_4_*a*_5_*a*_6_”) − 1} = {2, 9, 10,…, *n*_2_} ∩ {{4, 12, 98,…, *n*_3_}-1} ≠ Φ, then *P*_1_^1^ ⟶ *P*_3_^255^.

Similarly, *P* (“*a*_*n* − 4_*a*_*n* − 3_*a*_*n* − 2_*a*_*n* − 1_”) ∩ {*P* (“*a*_*n* − 3_*a*_*n* − 2_*a*_*n* − 1_a_*n*_”) − 1} ≠ Φ means *P*_*ik*−1_^*l*−1^⟶*P*_*ik*_^*l*^.

The *S* positional relationship is described as follows.

For each *S*, the decomposed sequence into a group of 4 can describe *P* {“AAAA”} = {3, 4,…, *n*_1_} for the “AAAA” sequence; there are a total of *n*_1_ positions in *S*; and *P* {“AAAC”} = {5, 2,…, *n*_2_} has a total of *n*_2_ positions in *S* for the “AAAC” sequence. Similarly, *P* {“TTTT”} = {14, 67,…, *n*_256_} has a total of *n*_256_ positions in *S* for the “TTTT” sequence. It can be seen that *P* {“AAAA”} + *P* {“AAAC”} + ⋯ + *P* {“TTTT”} = {3, 4,…, *n*_1_}+{5, 2,…, *n*_2_} + ⋯ + {14, 67,…, *n*_256_} = {1, 2, 3, 4,…,|*S*| − 3}; then, it can be described as *n*_1_ + *n*_2_ + *n*_3_ + ⋯ + *n*_256_ = |*S*| − 3.

**Theorem 2 .**

The DNA subsequence *T* can be decomposed into a group of 4 subsequences, and the subsequences describe the sequence *T* through the positional relationship:

(10) $$\begin{array}{c} P\left(i\right)=\left\{P_{1}^{i},P_{2}^{i},P_{3}^{i},...,P_{n}^{i}\right\},\;i=1,2,3,...,256. \end{array}$$

Among them, *P* (*i*) is the position information of the fourth quaternary combination, which refers to the position information corresponding to {*P*_1_^1^, *P*_2_^1^, *P*_3_^1^,…, *P*_*n*1_^1^}. Whether there is a correlation between any two *P* (*i*) and *P* (*j*), that is, *P*(*i*)⟶*P*(*j*), can be calculated as follows:

(11) $$\begin{array}{c} P\left(j\right)=P\left(i\right)-\left(j-i\right). \end{array}$$

Regarding whether the sequence *T* is a subsequence in *S*, *T* can be decomposed into the form of *T* = *P* (*n*_1_)*P* (*n*_2_) ... *P* (*n*_*i*_), if *P* (*n*_1_) has links with all *P* (*n*_*i*_). There are subsequences, namely,

(12) $$\begin{array}{c} P\left(n_{1}\right)=P\left(n_{i}\right)-4*n_{i},\;i=1,2,3,\ldots ,256. \end{array}$$

For example, *T* = “ACGAACCCCTAGAGACTAGCTAACCGGAATCAGCTA” is decomposed into *T* = *P* (7)*P* (6)*P* (93)*P* (115)*P* (113)*P* (91)*P* (14)*P* (46), and finally “A” is not considered. Among them, if the link of *P* (7)⟶, *P* (6)⟶, *P* (93)⟶, *P* (115)⟶, *P* (113)⟶, *P* (91)⟶, *P* (14)⟶, *P* (46) exists in S, then compare whether there is a link at the end of “A.” If the above process is established, it means that the sequence *T* is in the subsequence of *S* and the starting position of *P* (7) is the specific position of the subsequence *T* in *S*.

### 3.2. Mutation Detection Based on Position Index

The method of detecting mutation based on position index uses the correlation between positions to analyze whether there are mutation points in the sequence.

**Theorem 3 .**

If there are mutations such as SNP and InDel in the subsequence [25], the subsequence is decomposed into *P*(*i*)={*P*_1_^*i*^, *P*_2_^*i*^,…, *P*_*ni*_^*i*^}, *i* = 1, 2, 3,…, 256. If the subsequence exists in the decomposition, *P* (1) ⟶ *P* (2) ⟶ ⋯ ⟶ *P* (*i*) ↦ *P* (*m*) ↦ *P* (*j*) ⟶ ⋯ ⟶ *P* (*n*) means that the two cannot be directly connected but there is a correlation. The variation judgment formula (14) is as follows:

(13) $$\begin{array}{c} \left\{\begin{array}{cc} \text{SNP,} & \text{if }P\left[j\right]-P\left[i\right]=8,\\ \text{Insert,} & \text{if }P\left[j\right]-P\left[i\right]<8,\\ \text{Delete,} & \text{if }P\left[j\right]-P\left[i\right]>8. \end{array}\right) \end{array}$$

If *P* (1) ⟶ *P* (2) ⟶ *P* (*i*) ↦ ⋯ ↦ *P* (*j*) ⟶ *P* (*j +* 1) ⟶ *P* (*n*) forms two segments, when *P*(*j*) − *P*(*i*) ≫ 8, the positional relationship between the two is far greater than 8, and the two segments may belong to different genes. This variation is called structural variation. The local comparison algorithm is used for matching to determine the mutation position, and see the following:

(14) $$\begin{array}{c} \text{partial match}\left(P\left(m\right),\text{Substr}\left[T,P\left(i\right)+4,P\left(j\right)-1\right]\right). \end{array}$$

**Proof**

The following examples are used to illustrate the entire matching process, targeting the reference sequence *T* = “CATCCTCACTACCT,” decomposing *T* [*P* (1)] = “CATC,” *T*[*P* (2)] = “CTCA,” *T* [*P* (3)] = “CTAC,” normal matching *P* (1) ⟶ *P* (2) ⟶ *P* (3) is successful, indicating that there is a match between the sequences. If *P* (2) mutates, it becomes *P* (1) ↦ *P* (2) ↦ *P* (3).

If *P* (3) − *P* (1) = 8, SNP mutation occurs. Suppose the sequencing sequence becomes *S* = “CATCGTCACTACCT,” *T* [*P* (1)] = “CATC,” *T* [*P* (2)] = “GTCA” and Substr[*T*, *P*(1)+4, *P*(3) − 1], “GTCA” and “CATC” found the fifth position is caused by “C” mutation into “G.”

If *P* (3) − *P* (1) < 8, insert mutation occurs. Suppose the sequencing sequence becomes *T* = “CATCGCTCACTACCT,” *T* [*P* (1)] = “CATC,” *T* [*P* (2)] = “GCTC,” *T* [*P* (3)] = “ACTA.” Use *T* [*P* (2)] and Substr[*T*, *P*(1)+4, *P*(3) − 1], “GCTC” and “CTC” to find that “G” is inserted at the 5^th^ position.

If *P* (3) − *P* (1) > 8, delete mutation occurs. Suppose the sequencing sequence becomes *S* = “CATCTCACTACCT,” *T* [*P* (1)] = “CATC,” *T* [*P* (2)] = “TCAC,” *T* [*P* (3)] = “TACC.” Use *T* [*P* (2)] and Substr[*T*, *P*(1)+4, *P*(3) − 1], “TCAC” and “CTCAC” to find the fifth position and delete “C.”

Targeted sequencing is a method that refers to the sequencing of specific gene exon regions, with low cost and a sequencing depth of up to 1000. The exon regions of different cancer-targeted sequencing are different, and the raw data of targeted sequencing of different target regions are shown in Figure 8.

Figure 8 shows the sequencing data in two directions of the sequencing data. There are two files R1.fq and R2.fq, respectively. When the exon region is relatively short, the two sequences will overlap.

### 3.3. Position Optimization of Fast Learning Neural Network Based on Position Feedback

When a position index mismatch occurs in a position index relationship, there is no linear relationship between different positions, but most positions in the position index show a position similarity relationship, so it is necessary to introduce the position information into the feedback learning neural network for learning and determine whether there is a linear relationship between two or more position index relationships by inputting the position relationship, as shown in Figure 9.

## 4. Experimental Analysis of Targeted DNA Sequencing SNP Discovery Algorithm

### 4.1. Preexperiment Processing Flow

Since targeted sequencing is performed for specific gene exons, the sequenced sequence is shorter and the sequencing depth is deeper (the test depth is 1000). The range of the target sequence is shown in Table 1.

In Table 1, width is the sequencing width of the sequencer, which already includes the range of exons and some introns. The length of the illumina sequencing sequence is 150. Because it is paired-end sequencing, when the exons in the width are very short, paired-end sequencing will cause overlap. In Table 1, it is shown that the sequencing herein is flux-targeted DNA sequencing for 20 genes. The sequencing target region covers all coding regions of 20 genes, exon-intron junction (20–50 bp), and part of intron region of BRCA1/2 gene, with a total of 703 exon regions.

### 4.2. Sequence Alignment Software Read Quantity Comparison

In the early stage, the performance of Bowtie2 [26], BWA [27], Hisat2 [28], and Subread [29] was compared, and the number of comparisons was compared with the number of reads based on the location relationship matching algorithm. Count the number of reads of 703 exons, as shown in Table 2.

It can be seen from Table 2 that Posindex, based on the positional relationship indexing algorithm, has certain advantages in most exon regions. The BWA algorithm also performs quite well in the exon regions, and the worst effect is Hisat2. From Table 2, compare the average sequencing numbers of the exon regions of 20 genes, as shown in Figure 10.

It can be seen from Figure 10 that the Posindex algorithm has a clear advantage in the average number of exons in terms of statistics. In terms of gene CDH1 statistics, BWA, Subread, and Bowtie2 algorithms are better than Posindex algorithm; in terms of CHEK2, MAP3K1, and TLR4 statistics, Posindex algorithm is slightly inferior to BWA algorithm, better than Subread, Hisat2, and Bowtie2; in other gene penetrances, on the other hand, the Posindex algorithm has obvious advantages. Next, analyze the matching effect of the five algorithms from the overall matching rate of the number of reads. The matching rate is equal to the ratio of the number of successful matches in the target exon region to the number of matches in the Hg38 genome, as shown in Figure 11.

### 4.3. Comparison of SNP and InDel Variation Quantity

In the above comparison of commonly used algorithms, BWA software has the highest overall matching rate. Taking the Bam file generated by BWA as the research object, the mutation detection software packages Varscan2, GATK, Bcftools, and Freebayes were used to detect SNP and InDel and then compared with the location index detection algorithm to evaluate the performance. The common visualization software IGV [30] can view the variation of exon regions in bam files. The following table shows the number of SNP and InDel of exons, as shown in Tables 3 and 4.

In Table 3, the Posindex algorithm has certain advantages in terms of the number of SNPs, and the effect of Gatk is also ideal. Many SNP points are due to the lack of advantages of other software in terms of number, and the depth of sequencing will not meet the filtering requirements.

In Table 4, Gatk has an advantage in terms of quantity, but the variation points in Gatk do not exist statistically in other software, and false positives are relatively high. The Posindex algorithm is statistically reasonable.

Then, compare the number of SNP and InDel in the exon regions of 20 genes, as shown in Figures 12 and 13.

In Figure 12, the Posindex algorithm has a great advantage in the statistics of SNPs in exon regions.

In genes PTEN, CCND1, PALB2, and TOX3, other algorithms did not find SNP mutation points; on LSP1, BRCA2, BRIP1, STK11, BARD1, and MAP3K1 genes, the five types of algorithms have more SNP mutation points, and the Gatk effect is also ideal. Judging from the statistical number of SNP points in the overall gene region, the Gatk and Posindex algorithms are ideal in terms of detection effects, while the other three types of algorithms have average detection effects and similar numbers.

In Figure 13, the InDel detection quantity is similar to the SNP statistical quantity, and the Gatk and Posindex algorithm detection is ideal.

Compare the positions of the overall SNP and InDel with those of other software, and the effect is shown in Figures 14 and 15.

By analyzing the analysis process of SNP and InDel, the proposed method Posindex can find more mutation points, and the Gatk detection effect is also ideal, while Bcftools, Varscan2, and Freebyes detect fewer SNP and InDel mutation points. A high number of detection results does not mean a good detection effect, because there will be many false positives in the detection process, so the number cannot explain the detection advantage. The difference between Gatk and position index is that the false positive rate of Gatk is high, while the correct rate of position index is high.

The specific reasons are as follows:

1. In the original sequencing data, there are a large number of reverse sequences, containing a large amount of public data and index data, which cannot be completely deleted when cleaning up.
2. The problem of false negatives: there are many similar sequences in the DNA sequence, which may lead to relative sequencing data pointing to other locations. However, these sequences are not target sequences, resulting in a large number of false positives or false negatives, and many SNP and InDel mutation points will be lost.

## 5. Conclusion

In the detection of chemical genomic mutations, a DNA sequence matching algorithm based on the position index relationship is proposed to solve the problems of low accuracy and large differences in the detection of SNP and InDel mutations in the targeted sequencing sequence, which aims to establish the DNA sequence Position index relationship analysis SNP and InDel variation. First, divide the subsequence into *k* fixed sequences and establish links; secondly, analyze the position difference in the optimal link and establish a judgment model of position variation; finally, target the sequencing target area to cover the BRCA1/2 gene: the entire coding region, the exon-intron junction region (20–50 bp), and part of the intron region, a total of 703 exon regions. The actual data captured in the 101.3k area is used as an example to verify. The experimental results show that the location-based indexing method detects more mutation points than Bcftools, Freebyes, Vanscan2, and Gatk. After detecting SNP and InDel in this paper, it is found that the location-based index method has the best detection performance, but whether other data sets have the same effect needs a one-step test. Sequencing in other cancers will be applied and further analysis will be carried out later.

## Figures and Tables

**Figure 1:** Diagram of the fast learning network.

**Figure 2:** Diagram of feedback fast learning network.

**Figure 3:** Initialization matrix of the Needleman–Wunsch algorithm.

**Figure 4:** Effect picture of the Needleman–Wunsch algorithm after filling.

**Figure 5:** Needleman–Wunsch backtracking path.

**Figure 6:** Effect of global optimal ratio pair.

**Figure 7:** Path structure diagram based on location index topology diagram.

**Figure 8:** Original data structure of DNA targeted sequencing.

**Figure 9:** Feedback learning neural network index position relationship model.

**Figure 10:** Average number of gene exons.

**Figure 11:** Exon region matching rate.

**Figure 12:** SNP number in the gene region.

**Figure 13:** InDel number in the gene region.

**Figure 14:** Comparison of SNP position differences.

**Figure 15:** Comparison of InDel position differences.

**Table 1:** Target sequence range.

Number	Chr	Start	End	Width	Exon
1	chr2	214728618	214728776	159	BARD1
2	chr2	214728732	214728909	178	BARD1
3	chr2	214728870	28734619	177	BARD1
…	…	…	…	…	…
702	chr22	28734432	29126542	188	CHEK2
703	chr22	28734580	28734761	182	CHEK2

**Table 2:** Exon read number statistics.

Chr	Start	End	BWA	Subread	Bowtie2	Hisat2	Posindex
chr2	214728618	214728776	260	249	257	129	243
chr2	214728732	214728909	1064	1051	1055	579	1020
chr2	214728870	214729046	501	495	489	489	561
chr2	214730365	214730555	155	155	155	80	155
…	…	…	…	…	…	…	…
chr22	28730392	28730554	138	68	69	68	67
chr22	28734312	28734474	3247	3146	3215	1615	3207
chr22	28734432	28734619	4053	3908	2568	2024	3446
chr22	28734580	28734761	1126	559	560	560	1969

**Table 3:** SNP number in the exon region.

Chr	Start	End	Bcftools	Varscan2	Freebyes	Gatk	Posindex
chr11	1883898	1884084	0	1	1	0	1
chr11	108279407	108279546	1	0	1	0	1
chr11	108279497	108279656	1	0	1	0	1
chr5	56881868	56882067	1	1	1	1	1
chr5	56881992	56882186	1	1	1	1	1
...	...	...	...	...	...	...	...

**Table 4:** InDel number in exon region.

Chr	Start	End	Bcftool	Varscan2	Freebyes	Gatk	Posindex
chr11	1886659	1886816	1	1	1	1	2
chr11	1881380	1881555	1	1	1	1	1
chr11	1881456	1881639	1	1	1	1	2
chr13	32332572	32332740	1	1	1	2	1
chr13	32332576	32332740	1	1	1	2	1
...	...	...	...	...	...	...	...

## Data Availability

The raw data supporting the conclusions of this article will be made available by the authors, without undue reservation.
